The article "Machine Learning-Driven Enterprise Human Resource Management Optimization and Its Application" was retracted in 2023. Reasons: suspected computer-generated content; unreliable results or conclusions; concerns about the data; concerns about the results or conclusions.

# Machine Learning-Driven Enterprise Human Resource Management Optimization and Its Application

**DOI:** 10.1155/2022/2541421

**Published:** 2022-08-01

**Authors:** Jingtong Sun

**Affiliations:** ^1^Department of Management and Economics, Tianjin University, Tianjin, Nankai 300100, China; ^2^School of Economics and Management, Northeast Forestry University, Harbin, Heilongjiang 150001, China

## Abstract

With the advent of the Internet era, the frequency and proportion of candidates obtaining recruitment information through the Internet is getting higher and higher, and the amount of human resource information, such as talent information and job information, has also increased unprecedentedly, which makes human resource services face information overload. Especially with the gradual increase of the amount of information, this method is not enough for the acquisition and classification of massive data. After that, experts developed search engines to deal with the retrieval problem, and the first ones were Google and Baidu. As long as the search engine is clear about the direction of the search, it is indeed very convenient for the retrieval of massive data. However, in many cases, most users cannot clearly recognize the content they need or how to accurately express their needs. Faced with this problem, people propose recommender systems to solve the problem of obtaining preference information, which can better increase the user's experience and meet their own needs more easily. Based on the main workflow of the recommender system, this paper designs the overall architecture of the human resources recommendation system and implements a human resources recommendation prototype system based on deep learning. The system can better overcome the cold start problem and provide real-time recommendation results, improving the quality of HR personalized recommendation results.

## 1. Introduction

The development of the market has accelerated the competition among enterprises. The core competitiveness of an enterprise depends not only on sufficient capital and advanced technology but also on the human capital it has. To truly form capital, the human resources of enterprises must be effectively allocated and reasonably used. The maximum benefit of human capital can only depend on effective human resource management. Otherwise, it will only lead to increased internal friction, increased management costs, and brain drain. However, it is difficult to do a good job in human resources, and various management problems also occur from time to time, resulting in the dislocation between people and posts, resulting in a great waste of human capital. The first step of person post matching is to start from personnel recruitment. In the human resources industry, with the development of online recruitment, hundreds of millions of resumes and tens of millions of enterprise recruitment information have been accumulated through online recruitment channels. HR is faced with a large amount of unstructured data every day, such as various resumes, recruitment requirements of employers, and interview feedback reports. How to make efficient and full use of massive information has become the main focus of human resources for each company's department. Battlefield: with the development of enterprise information management, using information technology to improve the efficiency of enterprise management has become the consensus of contemporary enterprises. However, the inaccurate market positioning of enterprises and the lack of effective reflection of talent demand are also difficult problems in enterprise HR recruitment. In recent years, the rapid development of the Internet and information technology has eased many repetitive HR processes, such as ATS (automatic candidate management system), which greatly accelerated the interview process and facilitated the management of candidates. Another example is the salary management system, which makes the management of employees' personnel salary and social security simple and clear, but these are mainly process automation. It is very important to establish a perfect person post matching system. On the one hand, it helps enterprise recruiters find suitable candidates, and on the other hand, it also helps job seekers find suitable positions. In recent years, artificial intelligence technology has made great progress in speech recognition, image processing, semantic understanding, and other fields. These technological advances can help HR conduct preliminary candidate screening at the initial stage of personnel recruitment [1–8]. Therefore, this paper hopes to study and improve the recommendation algorithm based on deep learning and apply it to the field of human resources recommendation, in order to improve the current situation that the existing recommendation system using the algorithm is relatively traditional and single and at the same time improves the performance of the human resources recommendation system.

## 2. Related Work

In recent research, the recruitment big data enables researchers to conduct recruitment analysis in more quantitative ways. Among them, measuring the matching degree between talent qualification and post requirements, that is, the research of person post matching, has become one of the important topics. The early research work of person post matching can be traced back to the study by Malinowski and others. Using the file information of both candidates and jobs, they established a bilateral person post recommendation system to find a good match between talents and jobs. Subsequently, Lee et al. followed the idea of a recommendation system and proposed a job recommendation system for job seekers based on basic job preferences and interests. DSSM uses the convolution layer to extract semantic information for final prediction. Pjfnn initially proposed to take the person post matching problem as the classification task and take the “work resume” pair as the input to predict the matching degree. They proposed a joint representation learning method, which uses two convolutional neural networks (CNNs) to independently encode resume and position information and calculate cosine similarity as matching score. Using historical records, jrmpm uses a memory network to embed the preferences of candidates and recruiters into their representations. Recently, LightGCN proposed a graph convolution neural network to realize collaborative filtering, learning, comparing, and recommending the inner product of the embedded vectors of candidate nodes and task nodes. In fact, as an important task of enterprise recruitment, job matching has been well studied from different angles, such as job-oriented to measure skills, job seeker matching, and job recommendation. Along this line, some related tasks are also being studied, such as finding suitable talents and changing jobs. The “Internet+ industry” deeply integrates the Internet and traditional industries, and the industry's demand for talents is more accurate. Compared with the comprehensive recruitment model, the vertical recruitment model is smaller and more sophisticated, specializing in a certain field. The research on human resources recommendation at home and abroad is closely following the footsteps of recommendation algorithms, from machine learning to the current deep learning of the fire. Both at home and abroad, it analyzes user behavior data and obtains user job characteristics, so as to make job recommendations. . However, there are still problems similar to recommendation algorithms in today's human resources recommendation algorithm research. It still tends to recommend user preferences and behaviors. If users want to change jobs, they cannot be recommended at all. Therefore, the vertical recruitment model is a rapidly developing recruitment model in the future and will be more subdivided. The crowd is vertical or includes headhunters, students, blue collar workers, and programmers; industry vertical or includes finance, Internet, and medical treatment; and regional vertical or specific city recruitment. Social recruitment helps job seekers know more and more about the relevant information of the enterprise by establishing the social relationship between job seekers and employers, so as to judge the matching degree between the needs of the enterprise and their own situation [9, 10].

## 3. Related Theoretical Methods

### 3.1. Deep Learning

#### 3.1.1. Autoencoders

Autoencoder is a neural network model suitable for data compression, including encoder and decoder, as shown in the following figure. b is the output of encoder e after dimensionality reduction, and decoder d reconstructs the original input a from b by minimizing the loss function, thereby outputting c. Autoencoders are more suitable for training compression on data with similar datasets, and in the compression process, autoencoders perform lossy compression. Encoders and decoders are standard parametric equations, and in general, they are done using neural networks. When using optimization to minimize the loss function, the parameters of the encoder and decoder can be improved by, for example, stochastic gradient descent. Today, there are two main applications of autoencoders: denoising data and visualizing dimensionality reduction. Autoencoders can either cover relevant dimensions and distances, or learn data projections, as shown in Figure 1[11].

Autoencoders have the ability to capture complex relationships in raw data, as well as compact representations in hidden layers. On this basis, many excellent recommendation models have been proposed. These studies can be divided into two categories. The first category focuses on designing recommendation models based only on autoencoders without using any components of traditional recommendation models. However, these methods do not use any additional user and project information, which leads to the emergence of the second type of research. Its goal is to use the automatic coder to learn the intermediate feature representation and embed them into the classical collaborative filtering model. Collaborative filtering is improved by integrating the intermediate features of project entities into the matrix decomposition framework. The intermediate features are obtained by the automatic encoder. Because it unifies the weights of intermediate features to model, it may lead to limited improvement of model performance. In fact, each dimension of the intermediate features of different item entities obtained by unsupervised methods is predictable. Some feature elements contribute little to the prediction, and useless feature elements even introduce noise, which hinders the model.

#### 3.1.2. Contracted Autoencoder (CAE)

A systolic autoencoder is an unsupervised learning algorithm for generating useful feature representations. CAE can improve the robustness of the training dataset, and it differs from the autoencoder, in which a regularization term is added, the mapping has strong contraction in the training samples, and the encoder's mapping *f* has the norm of the Jacobian matrix of the input *x.* The number form is as follows:

(1) $$\begin{array}{c} J_{f\left(x\right)F}^{2}=\sum_{ij}{\frac{\partial h_{j\left(x\right)}}{\partial x\;i}}^{2}. \end{array}$$

The parameters of the autoencoder need to be learned by minimizing the reconstruction error and gradient penalty, and the cost function formula is as follows:

(2) $$\begin{array}{c} J_{\text{CAE}}\left(\theta \right)=\sum_{x\in D}\left(L\left(x,g\left(f\left(x\right)\right)\right)\right)+\lambda J_{f\left(x\right)F}^{2}, \end{array}$$

where *D* is the training set data, *L* is the reconstruction error, and *λ* is a hyperparameter that controls the regularization strength. CAE learns useful information through reconstruction error and shrinkage penalty. If reconstruction error needs to retain complete information, it needs to learn identity mapping. The shrinkage penalty makes the autoencoder reduce the dimensionality of the input information to a very small part. Both ways make most of the gradients of the input small, so when the input is less perturbed, the smaller gradient reduces those perturbations and improves the robustness of the encoder to small perturbations near the input [12].

### 3.2. Recommendation Algorithm

#### 3.2.1. Collaborative Filtering Recommendation Algorithm

Collaborative filtering is a classic recommendation algorithm, which is easy to implement and fast to calculate. Collaborative filtering algorithms are mainly based on similar users or items to recommend. The similarity between different users and posts can be achieved through various similarity formulas (such as cosine similarity). The basic assumption of this kind of algorithm is recommending their favorite items for users by finding other users with similar interest and preferences and then recommending the items they are interested in to the user. Collaborative filtering algorithms are mainly based on similar users or items to recommend. The similarity between different users and posts can be achieved through various similarity formulas (such as cosine similarity). As users use the site more frequently, more behaviors will be left behind, and there will be enough feedback information, so that the accuracy of predicting user behaviors will increase. Cosine similarity measures the angle between two vectors. In fact, the measure of cosine similarity is the magnitude of the cosine of the angle. When the two user vectors are calculated, the larger the cosine value, the more similar the two user vectors are, and the closer to zero. The similarity based on cosine distance characterizes the spatial angle relationship between different vectors, and the difference of positive and negative representing the direction is also different [13].

The Pearson coefficient is used to represent the correlation between user vectors, and its value range is [−1,1]. As with the similarity algorithm above, the larger the value, the higher the similarity. Based on the Euclidean distance, the absolute distance is calculated according to the coordinates of the point, which is suitable for calculating the similarity between symbols and Boolean values. Since the specific values of the two cannot be obtained, the final result can only be yes or no.

#### 3.2.2. Content-Based Recommendation Algorithms

Content-based recommendation algorithms are mostly used in text analysis research, such as news recommendation and advertisement recommendation. From the perspective of human resources recommendation, the content-based recommendation algorithm recommends jobs similar to the previous jobs to users based on their past jobs. Therefore, the core of content-based recommendation is to perform similar calculations on historical items. According to the content-based recommendation algorithm flow, items represented as application objects have many characteristics that can be described, and these characteristics can usually be divided into structural attributes and nonstructural attributes. Structure is a clear concept, and unstructured properties usually have vague meanings, no value constraints or can be used directly. For structured data, it can be used directly in algorithms in general, but when it comes to unstructured data like textual information, we often cannot model it before converting it into structured data.

#### 3.2.3. Recommendation Algorithm Based on Matrix Factorization

The principle of matrix factorization is to transform a rating matrix into several different feature matrices and multiply them. This method can simplify the matrix, and the subsequent recommendation algorithm calculates the decomposed matrix. In the raw data used by the recommender system, a large user rating matrix with *m* rows and *n* columns is usually formed. Taking the human resources user rating matrix as an example, *m* represents the number of job-seeker users, *n* represents the number of positions in the industry, the human resources user rating matrix is due to the scarcity of positions rated by users, a large number of positions have not been selected by users, and the data in the entire matrix is sparse. There will be a large number of vacancies in the matrix, and it is difficult to obtain the user's preference for the position according to the matrix, so it is difficult to improve the accuracy of the algorithm. The most primitive matrix decomposition is to decompose the user's rating matrix for the post into a multiplication of the user's and post's latent feature matrix. The matrix decomposition formula is as follows [14–16].

(3) $$\begin{array}{c} R_{m\times n}=U_{m\times d}\times W_{n\times d}^{T}. \end{array}$$

The matrix represents the user feature matrix, which represents the d-dimensional latent factor of user *u*, which is the internal characteristic of the user, and the matrix is the job feature matrix, which represents the d-dimensional latent factor of position *i*. According to the user feature matrix and post feature matrix in the above formula, the predicted score of user *u* for position *i* can be obtained as

(4) $$\begin{array}{c} y_{u,i}=u_{u}\times v_{i}^{T}. \end{array}$$

In some cases, the scoring matrix may not be decomposed into job-seeking user feature matrix and job feature matrix. It is necessary to continuously train the parameter theta by minimizing the deviation. By continuously adjusting the user feature matrix and the job feature matrix and calculating the predicted value. The difference from the true value is the predicted rating of job *i* by user *u*. (5) is the composition of the objective function L.

(5) $$\begin{array}{c} \text{theta}=\left(U,V\right), \end{array}$$

(6) $$\begin{array}{c} e_{u,i}=y_{u,i}-\hat{y_{u,i}}, \end{array}$$

The parameter theta is optimized using methods such as the least squares method to narrow the value between the predicted score and the actual score of the job-seeking user. When *L* is optimal, the most accurate prediction score can be obtained according to the obtained matrices *U* and *V*.

## 4. Design of Human Resource Management Optimization Algorithm System Based on Deep Learning

### 4.1. The Overall Structure of the System

The overall architecture of the human resources recommendation system is shown in Figure 2. In this paper, the recommendation system is divided into three layers, namely, the application layer, the middle layer, and the storage layer. The middle layer includes the data preprocessing layer and the recommendation calculation layer. The application layer, data preprocessing layer, and recommendation calculation layer are maintained by their respective subsystems, and the functions between the two layers are called through interfaces [17].

The application layer is developed using Java Web technology to provide interaction between candidates and the recommendation system. It is mainly divided into two parts: basic business applications and job recommendation applications. The basic business application of human resources includes functions such as applicant registration, login, job browsing, collection, and job application; job recommendation application includes personalized job recommendation and the latest popular job recommendation, which is responsible for the list of job positions recommended by the system to users presented to the user. For normal users, the system uses the results obtained by the recommendation calculation layer to make recommendations. When the logged-in user is a newly registered applicant, since the system does not have the user's predicted scoring information, the algorithm does not recommend the user at this time, and using the latest popular positions is recommended. The data preprocessing layer is implemented by the open source ETL tool Kettle, and its responsibilities include the following:

1. Data collection: collect user behavior log records from the application layer.
2. Building a data warehouse: cleans and transforms human resource data stored in business databases, builds a human resource data warehouse for HDCF algorithm processing, including cleaning and transforming user and item tables, analyzes and extracts behavioral data from log records, and constructs the scoring matrix, constructing a bag-of-words vector set of items.
3. Timely incremental update: use the Kettle tool to set timed tasks, regularly detect whether there is newly added candidate or job data in the business data table and synchronize the updated data to the data warehouse in time. When a new job posting is detected, a notification is sent to the recommendation computing layer.

The recommendation computing layer is the core of the human resources recommendation system, and its main responsibilities include (1) HDCF model training. The HDCF deep model is trained on the data in the data warehouse, and the predicted user-item rating matrix is obtained, which is used to provide personalized recommendations to the application layer; (2) the predicted rating matrix is updated online. After receiving the notification from the data preprocessing layer, the content-based filtering algorithm is used for the newly added post item, and its predicted score is obtained according to the basic attributes of the post and updated to the score matrix used to provide personalized recommendation; (3) the latest hot job statistics. Count the latest and most popular job postings and recommend them to newly registered candidates. The system calculates a priority weight for each job position (the weight is proportional to the number of visits to the job position and inversely proportional to the posted time of the job) and selects jobs with higher weights to form a recommendation set. The storage layer is the foundation of the recommender system and consists of MySQL and Redis. MySQL is used to store all the data in the recommendation system, including basic user data, job data, user behavior data, data warehouse for model training, and calculation results of the recommendation layer. Redis is used as a cache database to cache data such as prediction score matrix and latest popular recommendation list [18].

### 4.2. System Processing Flow

The basic processing flow of the human resources recommendation system is shown in Figure 3, which shows a series of workflows of the human resources recommendation system from data collection providing recommendation results to users. As can be seen from the data labels in Figure 3, the basic workflow of the recommender system includes the following five steps: (1) as shown in the data flow shown in label 1, the Java Web application provides basic business functions to candidates and shows the user a list of jobs recommended by the recommender system to the user. The ETL server collects the behavior log data of candidates in the process of interaction. (2) As shown in the data flow shown in labels 2∼3, the ETL server reads the original human resources data from the MySQL database, cleans and converts it, obtains the warehouse data for HDCF algorithm model training, and saves it to in a MySQL database. (3) As shown in the data flow shown in labels 4∼5, the recommended computing server reads the warehouse data from the MySQL database and performs two parts of computing work: one part is offline model training, and the predicted score matrix is obtained for personality. The other part is to calculate the latest popular weights of jobs and get the recommendation list of the latest popular jobs. After the calculation is completed, the recommended results to MySQL and the cache database Redis are saved. (4) As shown in the data flow shown in the label 6 ⟶ 4 ⟶ 5, The ETL server will regularly check whether there will be new jobs, so that the data can be updated in time to synchronize the Redis and MySQL databases. (5) As shown in the data flow shown in labels 7∼8, the system request sent by the Java Web application caches the corresponding business data from MySQL to the Redis database. At this time, Redis caches business data and recommendation calculation results and can efficiently respond to requests from applications.

## 5. Algorithm Evaluation and System Testing

### 5.1. Experimental Environment and Experimental Dataset

In this paper, experiments and analysis are carried out using real datasets. The data set used in this paper is the data collected from the human resources employment platform mentioned above. Through a series of data preprocessing work, a human resources data warehouse suitable for recommendation is obtained. The scale of the experimental data is shown in Table 1. The dataset contains 4692 candidates, 15000 jobs, and 170844 user behavior records. This results in the sparsity of the dataset:

The hardware and software environment of the system used in this experiment is shown in Table 2. The CDL and HDCF algorithms are implemented using the deep learning framework MXNet, the framework version is 0.8.0, built under the operating system Ubuntu Kylin 16.04 LTS, and the python version is 2.7.0.

### 5.2. Experiment Evaluation Metrics

There are five commonly used evaluation indicators for the currently commonly used recommendation algorithms, namely, MAE, RMSE, precision, recall, and F-measure. MAE and RMSE calculate the mean absolute error and mean square error of rating prediction. However, since the human resource recommendation set used in this paper only has behavior records of potential performance users and does not have the exact ratings of candidates for jobs, these two statistics are calculated. Indicators seem to be of little significance. In the human resources recommendation system, when a *R*_*ij*_ value in the user-item rating matrix is 0, it usually only means that the applicant *i* has not found the information of job *j* at all, but it cannot mean that he is not interested in job *j*. If the recommendation system recommends job *j* to it, it is not necessarily a wrong recommendation, so the accuracy rate cannot well reflect the performance of the recommendation algorithm. In this paper, for each user *i*, by sorting the predicted scores Ri of the items and recommending the top *N* items to the user, the recall rate recall@N for user *i* can be defined as

(7) $$\begin{array}{c} \text{recall}@N=\frac{\left|R_{i}\cap {\text{TRUE}}_{i}\right|}{\left|{\text{TRUE}}_{i}\right|}. \end{array}$$

Among them, *R*_*i*_ is the set of recommendation lists, and the size is *N*; TRUEi is the set of jobs, in which candidates are interested in, in the test set. In the human resource recommendation system, the smaller the *N*, the higher the recall rate, the better the performance.

### 5.3. Experimental Results and Analysis

The experiment in this paper divides the behavior records of candidates into two parts in chronological order, one part is the training set, accounting for about 90% of the total data, and the other part is the test set, accounting for 10% of the total data. Because the HDCF algorithm divides the human resource data into two parts, cold start and noncold start, and processes them with different algorithms. Here, the two parts of the data are briefly counted, and the results are shown in Table 3.

The experiment is divided into four parts: the parameter tuning of the deep model, the tuning of the deep network structure, the verification of the effectiveness of the algorithm, and the comparison of the algorithm effect. This section will introduce the experimental results and the conclusions of the analysis.

#### 5.3.1. Influence Experiment of Deep Model Parameters on Algorithm Performance

At the beginning of the experiment, this paper adopts the default settings of the CDL algorithm. Set *a* = 1, *b* = 0.01, *K* = 50, *w* = 1, *n* = 1000, *v* = 10, *u* = 1, batch_size = 256, and get the CDL and HDCF algorithms. The training process of the model is shown in Figure 4.

In Figure 4, the abscissa is the training time epoch of the algorithm model, and the ordinate is the target loss function value of the model. As can be seen from the curve in the figure, when the Epoch of the model training starts to reach 400, the CDL model basically converges, while the HDCF model basically converges, when the epoch reaches 500. Because the number of iterations required for an Epoch is as follows: number of samples/batch_size, and the number of iterations required for the two models to reach convergence is calculated. The CDL model is 400*∗*(15000/256)≈23500, and the HDCF model is 500*∗*(8791/256)≈17200. Therefore, this paper sets the number of iterations of the algorithm num_iter to 25000, at which time, both models can achieve the effect of basic convergence. At the same time, as can be seen from Figure 4, the absolute value of the loss function of the HDCF model is lower than that of the CDL model because the former only trains noncold-start projects, and the overall number of samples is less than the latter.

#### 5.3.2. Influence Experiment of Deep Network Structure on Algorithm Performance

The PMF module of the CDL algorithm defines the user and item latent semantic matrices as U and V, respectively, where the dimension of each latent semantic vector is K, and this K value is also the number of nodes in the coding layer of the PSDAE module, that is, the output of the low-dimensional coding. Number of dimensions: the K value represents the number of implicit features of users and items in the PMF algorithm. Appropriate K value is very helpful to improve the performance of the algorithm. Therefore, the influence of the latent semantic vector dimension K on the performance of the algorithm is experimentally tested and determined. The optimal K value and the experimental results are shown in Figure 5. As can be seen from Figure 5, with the increase of the latent semantic vector dimension K, the recall of the recommended results first increases and then decreases, indicating that the performance of the algorithm shows a trend of first increasing and then decreasing. The K value represents the number of hidden features in the human resources data. When the K value is small, the number of features extracted by the model is small, and the latent semantic vector is not enough to express the features of the data. At this time, increasing the K value can improve the performance of the algorithm. After the number of features extracted by the model reaches a certain level, increasing the K value at this time will reduce the performance of the algorithm. It can be seen from the figure that when the K value is 50, the recall rate of the CDL algorithm is the largest, and when the K value is 40, the recall rate of the HDCF algorithm is the largest, but it is close to the recall rate when the K value is 50. Subsequent experiments will set the latent semantic vector dimension K value to 50.

In addition, the main factor for judging the performance of the algorithm is to test the performance of the number of network layers in the deep network structure model. The experimental results are shown in Table 4.

Table 4 shows the recall rates of the two algorithm models when the number of network layers is 2, 4, and 6 layers, respectively. At this time, the encoder layers of PSDAE in the model are 1 layer, 2 layers, and 3 layers, respectively. It can be seen from Table 4 that when the number of network layers is 6, the recall rates of CDL and HDCF algorithms are the highest, and the recall rates of the two algorithms do not change much under 4-layer and 6-layer networks. Therefore, it can be judged that when the number of network layers reaches four layers, the ability of the PSDAE model to extract hidden features is relatively stable. Considering that the increase in the number of network layers brings a small recall rate gain, but it will lead to an increase in computational complexity, so the number of network layers is set to 4 layers.

## 6. Conclusion

The purpose of this paper is to study and improve the human resource management algorithm based on deep learning and apply it to the field of human resource management to improve the traditional and single status of the existing management system using the algorithm. With the help of the ability of deep learning feature extraction, this paper overcomes the main problems of traditional collaborative filtering algorithms such as data sparseness and cold start and improves the quality of human resource management. Collect the information of candidates and jobs from the human resources business system and then perform preprocessing operations such as cleaning, conversion, and reduction of the collected data, perform Chinese word segmentation and vectorization operations for the text fields, and finally obtain a management algorithm suitable for processed HR data warehouse. Based on the main workflow of the management system, the overall architecture of the human resource management system is designed, and a human resource management prototype system based on deep learning is implemented, which can better overcome the cold start problem and provide high real-time recommended results. The current algorithm implementation does not have enough scalability, so it is difficult to be competent for the analysis and processing of a large number of data in the real human resources system. In order to improve the practicability of human resources recommendation system based on deep learning and apply it in real business system in the future, we also need to try to implement HDCF algorithm on the distributed mxnet framework and design the distributed architecture of recommendation system based on deep learning [19, 20].

## Figures and Tables

**Figure 1:** Autoencoder architecture diagram.

**Figure 2:** Architecture of human resource recommendation system.

**Figure 3:** Workflow diagram of human resources recommendation system.

**Figure 4:** The training process of the CDL and HDCF algorithm models.

**Figure 5:** The recall rate recall@200 of CDL and HDCF under different K values.

**Table 1:** Human resources dataset size.

Name	Number
Applicants	4692
Jobs	15000
Behavior record	170844

**Table 2:** System software and hardware configuration.

Name	Value
CPU	Intel core i5-3350P CPU @3.10 GHZ × 4
RAM	16 GB DDR3 @1600 MHz
GPU	GeForece GT 620
Operating system	Ubuntu Kylin 16.04 LTS
Kernel version	GNU/Linux 4.4.0-53-generic x86_64
Python version	2.7.12
MXNet version	0.8.0 release

**Table 3:** Classification and statistics of human resources data.

Item category	Quantity	Quantity behavior record sheet in the test set
Cold start project	6209	1791
Non-cold start projects	8791	14790
All items	15000	16581

**Table 4:** Recall rate recall@200 under different network layers L.

Algorithm name	Number of network layers		
	2	4	6
SDL	0.5125	0.5509	0.5512
HDCF	0.5343	0.5725	0.5731

## Data Availability

The dataset can be accessed upon request.
